# Changes in the Quality of Life, Psychological Status, Medication Compliance, and Prognosis of Patients with Acute Myocardial Infarction after PCI by Applying PDCA Cycle Management Model

**DOI:** 10.1155/2021/7318653

**Published:** 2021-10-19

**Authors:** Yan Li, Mei Hong, Guohui Liu

**Affiliations:** ^1^Department of Cardiology, Renmin Hospital of Hubei University of Medicine, Shiyan, Hubei 442000, China; ^2^Department of Cardiothoracic Vascular Surgery, Renmin Hospital of Hubei University of Medicine, Shiyan, Hubei 442000, China

## Abstract

**Objective:**

To discuss the changes in the quality of life, psychological status, medication compliance, and prognosis of patients with acute myocardial infarction (AMI) after percutaneous coronary intervention (PCI) by applying plan-do-check-action (PDCA) cycle management model.

**Methods:**

A total of 125 patients with AMI who underwent PCI in our hospital from June 2018 to June 2020 were selected and divided into control group (*n* = 62) and research group (*n* = 63) by the random number method. The conventional nursing measures were used in the control group, and the PDCA cycle management model on the basis of the control group was used in the research group. The changes in the quality of life, psychological status, medication compliance, and prognosis were observed.

**Results:**

After intervention, the Generic Quality of Life Inventory-74 scores and the self-made medication compliance questionnaire score of the research group were higher than the control group (*P* < 0.05). After intervention, the self-rating anxiety scale score and self-rating depression scale score of the research group were lower than those of the control group (*P* < 0.05). The total incidence of adverse events in the research group (7.94%) was lower than that in the control group (20.97%) (*P* < 0.05).

**Conclusion:**

After the application of PDCA cycle management model, the quality of life, psychological status, medication compliance, and prognosis of AMI patients who underwent PCI were improved.

## 1. Introduction

Acute myocardial infarction (AMI) is acute myocardial necrosis caused by persistent coronary artery ischemia and hypoxia. Its main clinical symptoms include angina pectoris, chest pain, chest tightness, suffocation, upper limb numbness, dizziness, increased levels of serum markers of myocardial injury, and other performances [1]. AMI has an acute onset, rapid onset, and rapid progress. Patients can have myocardial injury and necrosis in a short time and even die in severe cases [2]. According to the survey, the incidence of AMI is high. In recent years, the global incidence of AMI has been increasing year by year, and the case fatality rate is as high as 5% to 8%, which poses a serious threat to the life and health of patients [3]. Percutaneous coronary intervention (PCI) is the most common and effective method for the treatment of AMI, which can fully unclog infarct-related arteries, restore effective myocardial perfusion, restore blood supply, and save myocardial function, which can significantly reduce mortality [4]. However, PCI surgery is not a one-time fix, and patients still need long-term followup treatment after PCI. PCI surgery may cause complications such as arrhythmia, nausea, and bleeding in patients with AMI, resulting in high levels of stress in the patient's body [5]. At the same time, because AMI patients lack systematic professional knowledge and require long-term rehabilitation after surgery, the patients are often accompanied by anxiety, depression, and other negative emotions, resulting in a huge psychological and spiritual burden for patients. Moreover, the medication compliance of AMI patients is often poor, which seriously affects the quality of life of AMI patients and adversely affects the prognosis [6]. Therefore, it is extremely important to provide high-quality and scientific nursing measures to AMI patients after PCI surgery.

The plan-do-check-action (PDCA) cycle management model was established by scholar Deming in 1954. It is a scientific concept that has been recognized by the public to solve the problem of work quality. The main feature of the PDCA cycle management model is to carry out quality management according to the order of plan (P), do (D), check (C), and action (A), so that the management objectives are gradually developed to achieve the final goal [7]. Studies have shown that the application of PDCA cycle management model in nursing quality management can greatly improve nursing quality and patient satisfaction [8]. This method not only takes the patient as the core but also proposes a targeted nursing plan based on individual differences and implements the nursing content. In addition, this method also carries out periodic feedback and summary in the nursing process, and then the nursing plan is adjusted in real time, so as to manage the patients' diseases in a circulative manner, which is conducive to reducing the missed items and promoting the patients' early recovery. It is time-sensitive and sequential [9]. Kong's team [10] conducted a study on 1020 patients receiving treatment in the endoscopy room, which included 512 patients in the PDCA group, and implemented a series of PDCA cycle management measures. The results found that, compared with the conventional management group, patients who applied the PDCA method had a lower incidence of nosocomial infections, sharp injury, and biological contamination and a higher rate of endoscopic cavity disinfection. This suggests that the PDCA cycle management to reduce the nosocomial infection rate, to prevent infection of cognitive aspects and so on, and to reduce the medical staff occupational exposure risk has a positive role. Chen's team [11] reported that the PDCA cycle method has good application value in the standardized nursing management of patients with severe COVID-19, which can effectively standardize nursing management and improve the survival rate of ICU patients.

In recent years, the PDCA cycle management model has been widely favored by physicians at home and abroad, but no research has been found to apply the PDCA cycle management model to AMI patients undergoing PCI surgery. Based on this, we observed the changes in the quality of life, psychological status, medication compliance, and prognosis of AMI patients undergoing PCI surgery after applying the PDCA cycle management model, in order to provide a certain reference for improving the quality of care.

## 2. Methods

### 2.1. Research Object

A total of 125 patients with AMI who underwent PCI in our hospital from June 2018 to June 2020 were selected and divided into control group (*n* = 62) and research group (*n* = 63) by the random number method.

#### 2.1.1. Inclusion Criteria

The inclusion criteria were as follows: ① all the patients were confirmed by coronary angiography and met the diagnostic criteria for AMI [12]; ② PCI was performed for the first time; ③ have an education level of primary school or above; ④ sign informed consent.

#### 2.1.2. Exclusion Criteria

The exclusion criteria were as follows: ① complicated with severe organ damage; ② complicated with other heart diseases; ③ complicated with malignant tumors; ④ patients with coagulation dysfunction; ⑤ patients with previous mental illness or cognitive behavioral abnormalities; ⑥ inability to followup; ⑦ patients who died during the study period.

### 2.2. Intervention Methods

#### 2.2.1. Control Group

The conventional nursing measures were used, a total of 6 months of intervention. Medical staff distributed brochures to AMI patients to explain the related knowledge of AMI and PCI, improved patient awareness of the disease, answered doubts, assisted patients to complete the examination, and corrected their bad living habits. When discharged from the hospital, the patient was again given health education, and the family members were asked to supervise the patient's medication, diet, exercise, etc.

#### 2.2.2. Research Group

On the basis of control group, the PDCA cycle management model was used, a total of 6 months of intervention. ① Plan: A PDCA cycle management and control team was established, with the head nurse as the team leader. All team members received professional training on AMI and PCI to ensure that each member was proficient in related nursing operations. Researchers used oral interviews or questionnaires to find out the current problems and causes of AMI patients. For example, patients were not familiar with the knowledge related to AMI, did not recognize the importance of correct self-management after PCI, had unreasonable diet, lacked exercise, were emotionally unstable, were easily agitated, forgot to take or missed taking drugs, and did not understand the serious consequences of not taking drugs. ② Do: Medical staff provided scientific and reasonable personalized health education for AMI patients after PCI and at the same time formulated health education intervention records form, including condition observation, medication guidance, diet guidance, activity guidance, sleep intervention, psychological counseling, rehabilitation guidance, discharge guidance, adverse event management, and other contents. Through timely communication with patients, nursing staff described the serious consequences of not taking medication, introduced the occurrence of adverse drug reactions, inquired about and recorded the medication status of patients, and analyzed the reasons for poor medication compliance of patients. Nurses should improve patients' cardiac function and prevent adverse cardiac events during hospitalization as the main prognostic goals, monitor patients' respiration, heart rate, consciousness, and other indicators, timely inform physicians to deal with abnormal conditions, and provide patients with continuous and intermittent low-flow oxygen inhalation and warm measures during the implementation of nursing. Medical staff established patient groups to share successful cases of treatment, encouraged patients to take the initiative in self-management, assessed the psychological status of patients, and used gentle language to comfort patients, thereby eliminating patients' negative emotions. Nurses monitored moderate exercise, told patients to get enough rest, told them to quit smoking and limit alcohol, and helped patients develop good habits. ③ Check: Under the leadership of the team leader, the researchers regularly supervised and examined the performance of patients and timely feedback of the improper nursing operation and analyzed the reasons for the poor prognosis of patients. Researchers closely observed the changes in patients' clinical symptoms and asked about and recorded their daily diet, exercise patterns and frequency, medications, and whether they had angina attacks. ④ Action: Researchers analyzed and summarized the results of inspections, actively searched for relevant factors that affect the effectiveness of nursing, paid attention to strengthening the improprieties in the nursing process, gave verbal encouragement to perform better behaviors, and enhanced the initiative of their participation; for poorly executed behaviors, they patiently analyzed the existing problems together with patients and revised and further rectified plans based on actual conditions, thereby promoting the next PDCA cycle management.

### 2.3. Research Tools

#### 2.3.1. Data Collection

Before the intervention and 6 months after the intervention, the researchers collected data from the two groups, and the second data set was collected by telephone to the clinic or door-to-door collection. The questionnaire was filled out by the research subjects on-site and collected on-site. The research subjects were guided by a uniformly trained researcher, who explained the research purpose and matters needing attention. If it was difficult for the patients to fill in the questionnaire by themselves, the researchers filled in the questionnaire instead, and the effective recovery rate of the questionnaire was 100%.

#### 2.3.2. Basic Information

The basic information questionnaire was designed by our hospital, including age, gender, location of lesion, complications during hospitalization, education level, marital status, and payment method of medical expenses.

#### 2.3.3. Quality of Life

The Generic Quality of Life Inventory-74 (GQOL-74) was applied, with 74 items including physical function, psychological function, social function, and life status. The total score of the inventory was 100 points. The higher the score, the better the quality of life. Cronbach's *α* of GQOL-74 scale was 0.885.

#### 2.3.4. Psychological States

① Self-rating anxiety scale (SAS): There were 20 items in total, and the 4-level scoring method was adopted, with 15 positive scores and 5 negative scores. <50 points indicate no anxiety, 50–59 points indicate mild anxiety, 60–69 points indicate moderate anxiety, and >69 points indicate severe anxiety. The higher the score, the worse the mental state. Cronbach's *α* of SAS was 0.924. ② Self-rating depression scale (SDS): There were 20 items in total, and the 4-level scoring method was adopted, with 10 positive scores and 10 negative scores. <53 points indicate no depression, 53–62 points indicate mild depression, 63–72 points indicate moderate depression, and >73 points indicate major depression. The higher the score, the worse the mental state. Cronbach's *α* of SDS was 0.919.

#### 2.3.5. Medication Compliance

The compliance of patients in the two groups was evaluated by the self-made medication compliance questionnaire based on the characteristics of the departments in our hospital. It mainly includes 4 questions: Do you take the medicine the number of times required by the doctor every day? Can you take the medicine as ordered by the doctor? Can you take the medicine regularly when requested by the doctor? Can you continue to take the medicine for a long time as required by the doctor after PCI? The 1–4 points' scoring method was used, which were completely impossible, mostly impossible, basically achievable, and completely achievable. The total score of the questionnaire was 16 points. The higher the score, the better the medication compliance. The content validity index of the self-made questionnaire in our hospital was 0.83, and internal consensus reliability Cronbach's *α* coefficient was 0.899, which has good reliability and validity.

#### 2.3.6. Prognosis

Six months after PCI, the incidences of postoperative adverse events such as angina, arrhythmia, heart failure, cardiac arrest, restenosis of myocardium, and revascularization were recorded in the two groups.

### 2.4. Statistical Analysis

Data were processed by the SPSS 22.0, measurement data was expressed as $\bar{x}$ ± *s*, and *t*-test was used for comparison. Count data was expressed as %, and *χ*^2^ test was used for comparison. Differences were considered significant at *P* < 0.05.

## 3. Results

### 3.1. The Basic Information between the Two Groups

There were no significant differences in age, gender, location of lesion, complications during hospitalization, education level, marital status, and payment method of medical expenses between the two groups (*P* > 0.05), as illustrated in Table 1.

### 3.2. The Quality of Life between the Two Groups

Compared with the situation before intervention, the GQOL-74 scores of the two groups were increased after intervention. After intervention, the gqol-74 scores of the research group were higher than those of the control group (*P* < 0.05), as illustrated in Figure 1.

### 3.3. The Psychological States between the Two Groups

Compared with the situation before intervention, the SAS score and SDS score of the two groups were reduced after intervention. After intervention, the SAS score and SDS score of the research group were lower than those of the control group (*P* < 0.05), as illustrated in Figure 2.

### 3.4. The Medication Compliance between the Two Groups

Compared with the situation before intervention, the self-made medication compliance questionnaire score of the research group was increased after intervention. After intervention, the self-made medication compliance questionnaire score of the research group was higher than that of the control group (*P* < 0.05), as illustrated in Figure 3.

### 3.5. The Prognosis between the Two Groups

The total incidence of adverse events in the research group (7.94%) was lower than that in the control group (20.97%) (*P* < 0.05), as illustrated in Table 2.

## 4. Discussion

AMI is a long-term ischemia and hypoxia in the patient's heart under the influence of many factors, resulting in myocardial cell necrosis, which has become a clinically frequent acute cardiovascular event. PCI can open infarct-related blood vessels and restore distal myocardial perfusion, which can directly and quickly relieve and improve blood vessel blockage and stenosis caused by atherosclerosis, so as to achieve smooth blood circulation and effectively improve myocardial ischemia. It is an efficient, safe, and minimally invasive treatment for AMI [13]. After PCI surgery, on the one hand, the physical function of AMI patients are impaired due to wounds, and stent implantation and balloon expansion can become stressors, causing patients to worry about their future quality of life. On the other hand, patients with AMI may worry about the stent falling off after the operation, and they are uncertain about the effect of the surgery, so they are prone to negative emotions such as psychological anxiety and depression [14]. Based on this, the implementation of high-quality nursing techniques for AMI patients after PCI plays a very important role in ensuring rapid recovery from the disease and improving the patients' living standards.

The PDCA cycle management model is a scientific nursing method derived from dynamic cycle management, through providing individualized nursing care for patients in a targeted manner and timely feedback to adjust in each link to make it change toward the expected goal, thereby shortening the recovery period, greatly improving the patients' satisfaction, and enabling continuous improvement in the quality of care. The PDCA cycle management model includes four stages, each stage is linked to each other, and the cycle is repeated, which can make nursing behaviors process integrated, professional, and standardized. In the continuous PDCA cycle, take the patient as the leading factor, repeatedly strengthen the patient's disease knowledge and skills in the process of problem solving, promote the spontaneous participation of the patient in self-disease management, and improve the overall level of care of the nursing staff, so as to guarantee patients' life safety [15].

### 4.1. Quality of Life

In this study, PDCA cycle management model was applied to AMI patients after PCI, and nursing measures were formulated in the whole nursing process according to the actual situation of the patients, and the plan was appropriately adjusted according to the individual's specific situation, through the physical and psychological states, living habits, and other aspects of nursing guidance, and a strict grasp of each specific nursing program, which is conducive to the standardization and scientization of the entire nursing procedure, to improve the trust and recognition of patients to nursing staff and accelerate the speed of rehabilitation to provide support. The PDCA cycle management model can improve the professional ability of nursing staff, standardize nursing procedures, and strengthen the ability of high-quality nursing execution, which plays an important role in improving the disease situation and postoperative quality of life of patients. In the planning stage, medical staff establish a good nurse-patient relationship with the patient through adequate communication with the patient, understand the patient's self-care ability, disease awareness, and medication compliance, and confirm the patient's actual care needs. In the doing phase, medical staff conduct scientific and reasonable health education for patients with AMI, prevent the occurrence of adverse cardiac events, share successful cases of treatment, and evaluate the psychological status of patients, so as to solve the problems existing in patients. In the checking and actioning stage, timely review of feedback and analysis and summary of deficiencies are conducive to timely correcting the patient's management misunderstandings, strengthening the norms of their own behavior, and promoting the entire nursing process to be carried out in an efficient and recurring manner. Therefore, AMI patients undergoing PCI have a high quality of life score [16].

### 4.2. Psychological Status

AMI patients undergoing PCI generally have various degrees of anxiety, depression, and other psychological conditions, especially after discharge, and wound infection and postoperative pain will aggravate the patient's anxiety. At the same time, after the operation, it is difficult for AMI patients to obtain professional nursing guidance, and the patients and their families lack the corresponding professional knowledge, which leads to the poor psychological condition of the patients. In this study, we found that, after applying the PDCA cycle management model, the SAS and SDS scores of AMI patients were decreased. The reason is that the PDCA method can enable patients to understand their own diseases and basic knowledge of PCI and avoid the fear caused by the unknown. In addition, by establishing patient groups to share successful cases of treatment, patients can learn from each other's experience, enhance patient initiative, and encourage patients to actively participate in rehabilitation after PCI. At the same time, medical staff evaluate the psychological condition of the patient and use gentle language to comfort the patient, which can relieve the patient's bad psychological state. The PDCA cycle management model focuses on the patient's physical and mental condition, which can greatly meet the needs of patients in various aspects such as physiology, psychology, society, and medication under personalized nursing and psychological care. It can improve the stress tendency of patients, provide more support to patients, and alleviate patients' bad emotions [17].

### 4.3. Medication Compliance

Some guidelines recommend long-term use of dual antiplatelet drugs for 9–12 months after PCI to reduce the incidence of vascular restenosis and stent thrombosis, so as not to affect the efficacy of PCI. It is necessary to continue antiplatelet therapy after PCI surgery, so as to improve the prognosis of patients. Studies have shown that there is a significant negative correlation between medication compliance and recurrence rate and mortality rate of patients with heart disease [18]. After discharge of AMI patients after PCI, due to various factors, postoperative health behavior execution is poor and medication compliance is low, which seriously affects postoperative recovery. Routine nursing is mainly based on the basic situation of patients after the implementation of basic nursing and can basically meet the physiological needs of patients. However, routine care suffers from formalization and lack of systematization and comprehensiveness, and infusion education is the mainstay, and patients are in a passive state. In addition, AMI patients are generally older, less receptive, forgetful, and poor in understanding, which leads to the poor effect of conventional care in improving patient's compliance with medications. The PDCA cycle management model performs cycle quality control on the basis of routine nursing services, formulates more detailed and specific nursing measures, and spirals upward to improve the quality of care, by communicating with patients in time, telling about the serious consequences of not taking medication, inquiring about and recording the patient's medication situation, giving timely feedback on the improprieties in the nursing operation, analyzing the reasons for poor medication compliance of patients, and carrying out the next cycle to improve the self-management of patients' medication. According to the characteristics of patients with AMI, medical staff provide medication guidance to patients in the form of telephone or face-to-face communication, so as to maximize the active initiative of patients in medication and improve medication compliance [19].

### 4.4. Prognosis

At present, there are many postoperative nursing measures for AMI patients undergoing PCI, but some patients have insufficient knowledge of the disease, lack of self-management ability, and simple nursing content, which will affect the prognosis of patients. PDCA cycle management model carries out orderly management of AMI patients after PCI through four systems; the spiral cycle can continuously improve the quality of care and control the risks in each stage. This will promote the improvement of patients' self-management ability, which may reduce the incidence of major adverse cardiac events after surgery. Medical staff use the PDCA method to strictly observe various clinical symptoms of AMI patients after surgery and to find out the relatively weak links of the patients through inspections, so as to carry out targeted and intensive education. At the same time, it analyzes the problems in the nursing process, defines the goals, implements the solutions, gives timely feedbacks on the improprieties in the nursing operation, and transfers the good methods and experience to the next round of PDCA cycle to form a repetitive feedback system. In the implementation of PDCA cycle management model, medical staff constantly eliminate potential risk factors in the nursing process by closely observing the clinical symptom changes of patients. In addition, AMI patients were informed of the PCI treatment process and the efficacy and treatment methods of complications in detail, and the postoperative required medications, medication methods, and adverse drug reactions were explained. This will improve the quality of care in a continuous cycle and have a positive effect on improving the prognosis of patients [20].

## 5. Conclusion

After the application of PDCA cycle management model, the quality of life, psychological status, medication compliance, and prognosis of AMI patients who underwent PCI were improved. The limitation of this study is that the number of the selected cases is small, and the patient's care efficiency is only evaluated in a short period of time. Therefore, it is necessary to carry out a large sample and long-term investigation in the future, which will have a positive effect on improving the quality of life of patients.

## Figures and Tables

**Figure 1:** The quality of life between the two groups. Compared with the status before intervention in the same group, ^*∗*^*P* < 0.05; compared with the control group after intervention, ^#^*P* < 0.05.

**Figure 2:** The psychological states between the two groups. Compared with the status before intervention in the same group, ^*∗*^*P* < 0.05; compared with the control group after intervention, ^#^*P* < 0.05.

**Figure 3:** The medication compliance between the two groups. Compared with the status before intervention in the same group, ^*∗*^*P* < 0.05; compared with the control group after intervention, ^#^*P* < 0.05.

**Table 1:** The basic information between the two groups (*n*, %).

Basic information	Control group (*n* = 62)	Research group (*n* = 63)	*χ* ^2^-value	*P* value
*Age (years)*				
40–59	29 (46.77%)	30 (47.62%)	0.009	0.925
≥60	33 (53.23%)	33 (52.38%)		

*Gender*				
Male	37 (59.68%)	35 (55.56%)	0.217	0.641
Female	25 (40.32%)	28 (44.44%)		

*Location of lesion*				
Extensive anterior wall	22 (35.48%)	21 (33.33%)	0.983	0.805
Partition wall	18 (29.03%)	20 (31.75%)		
Inferior wall	12 (19.35%)	15 (23.81%)		
High lateral wall	10 (16.13%)	7 (11.11%)		

*Complications during hospitalization*				
With	21 (33.87%)	19 (30.16%)	0.198	0.656
Without	41 (66.13%)	44 (69.87%)		

*Education level*				
Primary school	27 (43.55%)	25 (39.68%)	0.427	0.935
Junior high school	19 (30.65%)	22 (34.92%)		
High school or technical secondary school	10 (16.13%)	11 (17.46%)		
College degree or above	6 (9.68%)	5 (7.94%)		

*Marital status*				
Married	47 (75.81%)	50 (79.37%)	0.228	0.633
Widowed/divorced/unmarried	15 (24.19%)	13 (20.63%)		

*Payment method of medical expenses*				
Medical insurance	36 (58.06%)	34 (53.97%)	0.213	0.645
Rural cooperative medical service	26 (41.94%)	29 (46.03%)		

**Table 2:** The prognosis between the two groups (*n*, %).

Group	Angina	Arrhythmia	Heart failure	Cardiac arrest	Stenosis of myocardium	Revascularization	Total
Control group (*n* = 62)	5 (8.06%)	3 (4.84%)	2 (3.23%)	1 (1.61%)	1 (1.61%)	1 (1.61%)	13 (20.97%)
Research group (*n* = 63)	2 (3.17%)	1 (1.59%)	1 (1.59%)	0 (0.00%)	1 (1.59%)	0 (0.00%)	5 (7.94%)
*χ* ^2^-value	—	—	—	—	—	—	4.305
*P* value	—	—	—	—	—	—	0.038

## Data Availability

The data used and/or analyzed during the current study are available from the corresponding author.
